The article "Impacts of Groundwater Discharge at Myora Springs (North Stradbroke Island, Australia) on the Phenolic Metabolism of Eelgrass, Zostera muelleri, and Grazing by the Juvenile Rabbitfish, Siganus fuscescens" was published in 2014. Journal: PLoS One.

# Impacts of Groundwater Discharge at Myora Springs (North Stradbroke Island, Australia) on the Phenolic Metabolism of Eelgrass, *Zostera muelleri*, and Grazing by the Juvenile Rabbitfish, *Siganus fuscescens*

**DOI:** 10.1371/journal.pone.0104738

**Published:** 2014-08-15

**Authors:** Thomas Arnold, Grace Freundlich, Taylor Weilnau, Arielle Verdi, Ian R. Tibbetts

**Affiliations:** 1 Biochemistry and Molecular Biology program, Dickinson College, Carlisle, Pennsylvania, United States of America; 2 School of Biological Sciences, The University of Queensland, Brisbane, Australia; Università della Calabria, Italy

## Abstract

Myora Springs is one of many groundwater discharge sites on North Stradbroke Island (Queensland, Australia). Here spring waters emerge from wetland forests to join Moreton Bay, mixing with seawater over seagrass meadows dominated by eelgrass, *Zostera muelleri.* We sought to determine how low pH / high CO_2_ conditions near the spring affect these plants and their interactions with the black rabbitfish (*Siganus fuscescens*), a co-occurring grazer. In paired-choice feeding trials *S. fuscescens* preferentially consumed *Z. muelleri* shoots collected nearest to Myora Springs. Proximity to the spring did not significantly alter the carbon and nitrogen contents of seagrass tissues but did result in the extraordinary loss of soluble phenolics, including Folin-reactive phenolics, condensed tannins, and phenolic acids by ≥87%. Conversely, seagrass lignin contents were, in this and related experiments, unaffected or increased, suggesting a shift in secondary metabolism away from the production of soluble, but not insoluble, (poly)phenolics. We suggest that groundwater discharge sites such as Myora Springs, and other sites characterized by low pH, are likely to be popular feeding grounds for seagrass grazers seeking to reduce their exposure to soluble phenolics.

## Introduction

North Stradbroke Island (NSI) is one of the world's largest sand islands, covering 285 km^2^ and framing the east side of Moreton Bay in southeast Queensland, Australia. The island, also known by its aboriginal name of Minjerribah, is surrounded by extensive seagrass meadows [1], [2] which are grazed by fishes, turtles, and dugongs and serve as nursery grounds for other native species (e.g., [3]–[6]).

The unusual geomorphology of NSI allows rainwater to recharge a massive aquifer of groundwater, forming a “central mound” or lens of freshwater under the island [7]. Pressure within this aquifer prevents saltwater intrusion and drives groundwater out beyond the coastline and into numerous creeks, swamps, window lakes, and springs on the island. One such release point is Myora Springs, located on the west coastline of NSI. Myora springs discharges approximately 2.4 million liters day^−1^ of groundwater through a mangrove forest and paperbark (*Melaleuca quinquinervia*) swamp and into Moreton Bay [8]–[10]. Here spring waters mix with seawater over shallow seagrass meadows dominated by eelgrass, *Zostera muelleri.* The degree of mixing is dependent upon the tides; for at least several hours per tidal cycle, at low tide, the effluent extends over 2500 m^2^ of exposed seagrass meadow. Several observations suggested that spring effluent might be impacting the shallow water marine community at this site; for example, anecdotal reports from local fisherman describe pitted and eroded shells in this area and we observed a lack of calcareous epiphytes on seagrasses near the shoreline, both of which suggest possible low pH conditions [11]. Indeed, a preliminary study in January 2012 revealed that spring effluent, pH 5, extended over exposed seagrass meadows during low tides, depressing seawater pH by ∼0.5 units at a distance of 10–20 m from the edge of the mangrove forest, without detectable changes in salinity at this distance.

Previously we found that low pH conditions and the corresponding increases in seawater CO_2_ levels were associated with a dramatic loss of protective phenolic substances, including phenolic acids and condensed tannins, in four different populations of seagrass ([12], also see [13]). These results were surprising since terrestrial plants exposed to elevated CO_2_ conditions often exhibit *increased* levels of many ‘carbon-based’ secondary metabolites, including (poly)phenolics [14]–[21]. Indeed, light and carbon availability stimulate the shikimic acid and phenylpropenoid (SA/PP) pathways that synthesize most plant phenolics [22]–[24]. Whatever the cause, such a loss of seagrass phenolics may have ecological consequences; they serve as herbivore deterrents, digestion reducers, and antifoulants and some possess antimicrobial properties, inhibiting the growth of the marine pathogen *Labyrinthula* which causes the seagrass wasting disease [25]–[37].

In the earlier set of experiments [12] the potential impacts on herbivores were not investigated because there were few important seagrass grazers at those study sites. In contrast, there are numerous large herbivores consuming significant quantities of seagrass in Moreton Bay. Here we sought to determine how the spring affects the dominant macrophyte *Z. muelleri* and interactions with one co-occurring grazer, the black rabbitfish (*Siganus fuscescens*).

## Methods

### Study Site

Myora Springs is located on the west coast of North Stradbroke Island, Queensland, Australia (7°30′54.7″S 153°27′43.5″E). It is one of many island habitats, including creeks, gullies, swamps, and perched lakes, receiving freshwater from a pressurized lens of groundwater [8], [9]. In this case spring water flows through several types of forested wetlands, including a paperbark swamp, eucalypt woodland, and mangrove forest, before reaching Moreton Bay [10]. Preliminary surveys, conducted at low tide, suggested that spring waters flowing westward onto exposed seagrass meadows, mixed with seawater from Moreton Bay to generate a pH gradient. We examined seagrass patches along this gradient, focusing on areas located 5–10 m (near spring) and 30–50 m (background) from the spring outflow which differed in pH but not salinity during low tides (Fig. 1).

**Figure 1:** Spring water from Myora Springs emerges from a mangrove forest (A) and discharges over shallow seagrass beds in Moreton Bay, Australia, during low tides (B). Shoots of *Zostera muelleri*, collected from “near spring” sites 5–10 m from the mouth of the spring and “background” sites at distances of 30–50 m were used in pair-choice feeding trials. Clusters of shoots from each location (C) were offered as food items to juvenile black rabbitfish, *Siganus fuscescens* (D).

### Water analyses

Preliminary analyses of the site were conducted in March and April 2012 using handheld instruments [12]. In April 2012 a series of discrete water samples from the spring itself and additional “near spring” and “background” sites were collected. Samples were immediately transported on ice to SGS Environmental in Rocklea, Queensland (NATA accreditation #2562, site 2070) for analysis of pH, alkalinity, total nitrogen, total Kjeldahl nitrogen, nitrates, nitrites, and sulfates. Corresponding pCO_2_ values were calculated using the CO2SYS 1.05 program [38], [39] with constants of Cai and Wang [40].

### Specimen collections

The collection of juvenile black rabbit fish, *Siganus fuscescens*, was conducted by nighttime seining in One Mile Harbor, Dunwich under the auspices of permit SBS/182/12/URG/GOODMAN FOUNDATION to I.R. Tibbetts. Fish were held overnight following the animal care policies of Queensland Animal Care and Protection Act 2001 (Animal Care and Protection Regulation 2012) in shaded tanks supplied with fresh seawater from the seawater system at the Moreton Bay Research Station (MBRS), University of Queensland as approved by the institution's Institutional Animal Care and Use Committee (IACUC). *Zostera muelleri* was collected from Myora Springs site under the auspices of permit #QS2011/MAN151 from the Queensland Department of Environment and Resource Management awarded to T. Arnold. Collections were made at ten “background” sites, located 30–50 m from the spring outflow, and ten “spring” sites located 5–10 m from the mouth of the spring. Plants were immediately transported in cool dark insulated containers, between layers of seawater moistened towels, to MBRS.

### Feeding experiments

For feeding trials, blades from shoots of *Z. muelleri* were gently wiped clean of fouling organisms and clipped to consistent 10 cm lengths. Three to five shoots, each possessing 3–4 blades were fastened together, weighed, and affixed at one end to plastic tubes filled with sand, to mimic the morphology and orientation of intact eelgrass shoots (Fig 1c). The average mass for these clusters of eelgrass shoots was 0.85 g wet mass (WM). Similar sections, and bulk plants, were stored at −80°C and subsequently transported to Dickinson College, Carlisle, PA (USA) encased in dry ice. Paired choice feeding trials were conducted in a series of 12 shaded 50 liter tanks containing four juvenile rabbitfish each (Fig 1d). Fish had been acclimated to tanks and had not had access to food for 24 hours prior to the trials. Weighted groupings of seagrass shoots, one from “background” sites and one from “near spring” sites, were placed into randomly selected ends of each tank at the start of the trials. Trials concluded when one food item was ∼50% consumed; clumps were removed, blotted dry, weighed and measured. Each fish participated in only 1 trial. To control for potential non-grazing weight loss a set of seagrass food items (n = 3 from both sites) were placed into similar tanks without fish for corresponding time periods [41]. We observed no autogenic loss of tissue for these controls.

### Tissue analyses

Analyses of seagrass metabolites were conducted for leaf tissues (without roots and rhizomes) harvested from each location. Leaves were gently wiped clean of epiphytes. For elemental analyses second and third rank leaves from four *Z. muelleri* plants per location were combined, dried, and homogenized. Samples (3–5 mg each) were analyzed for carbon and nitrogen contents as well as ^13^C and ^15^N signatures on a Europa isotope ratio mass spectrometer at the Stable Isotope Laboratory at the University of California Davis. Biochemical analyses were conducted on tissues samples stored at −80°C. Leaf tissues for 3–5 shoots per location were homogenized using a HT high throughput grinder and extracted in MeOH(aq) with 2% acetic acid (except in the case of phenolic acid analyses) for 24 h at 4°C in the dark. Concentrations of phenolic acids were determined by RP-HPLC using a gradient method modified described previously [12], [42]. Fifteen µl of each extract were injected onto an Agilent Eclipse Plus RP-18 HPLC column. Phenolic acids previously attributed to *Z. muelleri* [42] were identified by comparison to commercial standards and concentrations (mg compound g^−1^ blade DM) determined using individual standard curves. Condensed tannins (proanthocyanindins) and Folin-reactive phenolics were quantified using micro-plate assays derived from the acid-butanol and micro-Folin methods [43]–[46] with standard curves developed using quebrancho tannin obtained from A. Hagerman (Miami University of Ohio) and gallic acid (Sigma), respectively. Natural product concentrations were expressed as mg compound g^−1^ tissue wet mass (WM) or %WM. Lignin contents were determined for *Z. muelleri* shoots from 10 locations. Five to eight shoots per location were cleaned, pooled, air-dried, and homogenized. Well-mixed 75 mg aliquots were analyzed using the methods of Foster et al [47]. Acetyl bromide soluble lignin (%ABSL) was calculated using the coefficient 17.75 and expressed as mg g^−1^ cell wall unit.

### Statistical analyses

Statistical analyses were conducted using SigmaStat. Datasets comparing two groups were analyzed using two-tailed Student's t-tests or Mann-Whitney Rank Sum Test with an α level of 0.05. Water chemistry data and datasets resulting from the analyses of tissues from previous experiments (see [12]) which examined three sampling sites groups were compared using ANOVAs with Holm-Sidak multiple comparisons or, when transforming data did not satisfy test assumptions, with Kruskal-Wallis One Way Analysis of Variance on Ranks with Tukey or Dunns multiple comparisons.

## Results

We observed that for the common seagrass *Z. muelleri* proximity to Myora Springs was associated with increased grazing by juvenile black rabbit fish and a dramatic and nearly complete loss of soluble phenolics, such as phenolic acids and condensed tannins, but not insoluble lignins.

### Site characterization

As expected, the spring effluent was cool, fresh, and relatively acidic. The spring was not a significant source of alkalinity, sulfates, total Kjeldahl nitrogen and nitrite but did contain elevated levels of nitrate (Table 1). During low tides the effluent extended over the exposed seagrass meadows, over an area of ∼2500 m^2^, mixing with Moreton Bay seawaters. The plume of spring water influenced seawater chemistry 5–10 m from the source; here, pH was depressed an average of 0.5–0.8 units and corresponding pCO_2_ values were increased ∼400%, reaching an average level of 1749 ppm (Table 1). Spring water dilution of seawater resulted in slightly lower levels of sulfates, total Kjeldahl nitrogen, and total N, compared to unaffected sites located 30–50 m away (Table 1). At this distance, we observed no significant reductions in salinity or water temperatures, during low tides. *Zostera muelleri* was the dominant seagrass, with *Halophilla ovalis* interspersed. The presence of shallow channels of spring water near the shore and occasional ∼1 m diameter depressions in the sediment (stingray feeding sites) generated some patchiness within an otherwise dense seagrass meadow. Except for the aforementioned differences in epiphytic cover seagrasses from the various sites were indistinguishable. We did not observe signs of grazing (e.g. bite marks) on *Z. muelleri* leaves. However, this is not surprising since most co-occuring herbivores, including rabbitfish, tend to consume whole blades or shoots, without leaving tell-tale grazing scars.

**Table 1:** Chemical characteristics of water near Myora Springs, North Stradbroke Island, Australia in April 2012.

Conditions	Seawater chemistry				
Distance from seep	Spring	5–10 m	30–40 m	Test	P
Temperature (°C)	23.15±0.66^a^	24.92±0.16^ab^	26.56±0.97^b^	1	**0.019**
Salinity	2.7±0.8^a^	35.3±0.2^b^	35.4±0.3^ b^	2	**0.009**
Total Kjel. Nitrogen (calc) (mg/L)	0.117±0.003^a^	0.192±0.039^ab^	0.287±0.024^b^	1	**0.021**
Alkalinity - Total as CaCO_3_ (mg/L)	<2^†^	120.0±0.0	120.0±0.0	2	**0.071**
Nitrate as N (calc) (mg/L)	0.117±0.009^a^	0.049±0.014^b^	0.001±0.001^c^	1	**0.001**
Nitrite + Nitrate as N (mg/L)	0.120±0.006^a^	0.054±0.014^b^	0.002±0.001^c^	1	**0.001**
Nitrite as N (mg/L)	0.004±0.000	0.005±0.001	0.005±0.000	1	**0.706**
Total Nitrogen as N (mg/L)	0.237±0.003	0.248±0.026	0.307±0.024	1	**0.136**
Sulphate as SO_4_ (mg/L)	2.6±0.3^a^	1937.5±531.3^ab^	2566.7±120.2^b^	2	**0.023**
pH Value @25°C	5.5±0.1^a^	7.8±0.3^ab^	8.5±0.0^b^	2	**0.001**
pCO_2_ (µtm)		1749±157^a^	572.4±0^b^	3	**0.002**

Statistical analyses: 1, one-factor ANOVA with Holm-Sidak multiple comparisons; 2, Kruskal-Wallis One Way Analysis of Variance on Ranks with Tukey or Dunns multiple comparisons; Student's t-test. ^†^below detection limit, did not test.

Values are means +/− SE.

### Feeding experiments

Rabbitfish began to consume *Z. muelleri* immediately and most feeding trials were completed within 30 minutes, when ∼50% of the “near spring” tissue mass had been consumed. *S. fuscescens* fed preferentially upon seagrass blades collected near the spring (Figure 1; Mann-Whitney Rank Sum Test, P = 0.012). A total of 48 fish, from twelve replicate aquaria, consumed significantly more “near spring” tissue (55% or an average of 400 mg tissue trial^−1^), compared to tissue from plants collected at “background” sites (25% or an average of 200 mg mg tissue trial^−1^).

### Elemental analyses

Neither the carbon and nitrogen contents nor the C:N ratio of seagrass foliage were significantly altered by proximity to the spring (Table 1). The δ^13^C and δ^15^N signatures of plant tissues were both significantly increased near the spring (Student's t-test; P = 0.001 and P = 0.003, respectively). These values and the observed increases are similar to previously reported isotopic signatures for *Z. muelleri* on NSI [48].

### Biochemical analyses

We found that *Z. muelleri* from sites >30 m from the spring outflow accumulated significant levels of proanthocyaninidins (condensed tannins) and possessed many, but not all, of the expected phenolic acids previously reported for this species (see [41]). The concentrations of all soluble phenolics decreased significantly, often becoming undetectable in plants sampled within 5–10 m of spring. For example, concentrations of total reactive phenolics, measured by the Folin assay, dropped 87% (Fig. 3, Student's t-test, P<0.001). Similarly, foliar concentrations of condensed tannins dropped from an average of 15.5% DM, a relatively high value for this seagrasses, to essentially undetectable in *Z. muelleri* exposed to the spring effluent (Fig. 3, Mann-Whitney Rank Sum Test, P<0.001). Levels of the predominant phenolic acids, gallic acid and rosemarinic acid, were all significantly lower; in fact, near the spring effluent only 7% and <1%, respectively, of these compounds remained (Student's t-test, P = 0.001 and Mann-Whitney Rank Sum Test, P = 0.008). Caffeic acid levels were undetectable in most plants regardless of location. Acetyl bromide soluble lignin contents of the leaf tissues collected from near spring locations in April 2012 were not significantly different compared to “background” samples collected 30–50 m away (Fig 3, Student's t-test, P = 0.586). Given our past observations we anticipated that conditions near the spring would alter lignin levels. To confirm that they do not we conducted additional analyses of *Z. muelleri* tissues collected from the same sites in March 2014. As before, we detected no difference in leaf lignin contents (Fig 3, Student's t-test, P = 0.932).

## Discussion

Myora Springs surface water flowing through paperbark and mangrove forests was low in salinity, alkalinity, pH, total and Kjeldahl N, and sulfates but higher in nitrates, compared to Moreton Bay seawater (Table 1). At the coast, spring water mixed with seawater, generating a gradient of abnormally low pH conditions within a ca. 2500 m^2^ area during low tides. The pH of seawater over emergent seagrasses was reduced by ∼0.7 units; for example, in early April we observed pH 7.8 waters at sites within 10 m of the effluent, compared to an average of pH 8.5 for seawater collected 30–50 m away. Similar conditions were recorded throughout March and April 2012. Most other conditions were unaffected, or affected to a minimal degree. Eelgrass shoots collected near the outflow of the spring were apparently healthy and, except for a lack of calcareous epiphytes, indistinguishable from plants collected 30–50 meters away.

Seagrass proximity to the spring altered the feeding behavior of a native grazer, the black rabbitfish, *Siganus fuscescens*. In paired-choice feeding trials juvenile rabbitfish immediately identified and preferentially consumed *Zostera muelleri* leaves collected nearest to the spring. They removed approximately twice the tissue from these plants, in terms of total mass and percent mass lost, compared to those collected from more distant sites (Fig 2). In fact, they often ignored seagrasses collected from more distant sites until much of the other, more preferred leaves were consumed.

**Figure 2:** Results of paired-choice feeding trials for juvenile black rabbitfish, *Siganus fuscescens*, feeding on eelgrass, *Zostera muelleri*. Food items collected from multiple locations 5–10 m (open bar) and 30–50 m (filled bar) from the outflow of Myora Springs, North Stradbroke Island, Australia. Bars represent the mean of 10 trials each, with ±SE error bars.

**Figure 3:** Results of chemical analyses for above-ground tissues of eelgrass, *Zostera muelleri*, collected from multiple locations 5–10 m and 30–50 m from the outflow of Myora Springs, North Stradbroke Island, Australia. Bars represent the group means, with ±SE error bars. *indicates P<0.05.

The feeding preferences of marine grazers, including fishes, can often be influenced by seagrass carbon and nitrogen contents which, in turn affect leaf toughness and digestibility [49]–[52] but this did not seem to be a factor in our feeding trials simply because these characteristics did not differ significantly in the seagrass leaves from the two locations. For example, nitrogen input from Myora Springs was relatively low, even though nitrates were elevated, and we did not detect a significant change in *Z. muelleri* tissue %N near the spring (Table 1). The %N contents and ^15^N signatures we observed for *Z. muelleri* tissues were comparable to values reported for relatively other un-impacted sites in Moreton Bay [48]. The small change in tissue ^15^N signatures near the spring may indicate some limited input of anthropogenic nitrogen [48], [53] but this did not alter the nitrogen content of the seagrasses (Fig. 3) Similarly, we found that carbon contents of *Z. muelleri* tissues were not altered significantly by proximity to spring effluent. This was surprising since *Z. muelleri* the estimated pCO_2_ concentrations were elevated ∼400% near the spring, at least during low tides. Leaf δ^13^C signatures suggested that carbon assimilation had been enhanced in the recent past, as would be expected for plants possessing poor carbon concentrating mechanisms (e.g., [54]–[56]) at these high CO_2_ locations (Fig. 3). As the unaltered %C and %N contents would suggest, seagrass tissue C:N ratios were unchanged. They were similar to those reported for this species in nearby locations [53].

To determine if it is common for seagrass C and N contents to be unaffected by high CO_2_ / low pH conditions we analyzed tissues from a previous study examining the response of other seagrass species at Mediterranean CO_2_ vents sites and in free ocean carbon enrichment experiments [12]. These results were indeed similar: low pH / high CO_2_ conditions did not alter carbon and nitrogen contents, carbohydrate levels, or protein contents in these earlier studies (Tables 2,3; see [12] for site descriptions). Similarly, C:N ratios from these earlier studies did not change, or change in any particular direction. We detected similar decreases in the δ^13^C values of *Cymodocea nodosa* growing near this high CO_2_ vent near the island of Vulcano, Italy which is consistent with the previous reports of Vizzini et al [56] who detected a similar decrease in δ^13^C values of *Posidonia oceanica* exposed to high CO_2_ vents near Panarea, Italy.

**Table 2:** Composition of *Cymodocea nodosa* shoots collected at various distances from the natural CO_2_ vent site from the Island of Vulcano, Italy in 2011 and 2013.

Conditions	Seawater carbonate chemistry^†^		
Distance from seep	380 m	300 m	260 m
Salinity	37.16±0.07	37.12±0.06	37.05±0.1
pH (units)	8.11±0.01	7.84±0.04	7.32±0.05
pCO_2_ (µtm)	422±43	976±269.5	4009±1442.7
TA (µmol kg^−1^)	2549.6±29.6	2555.9±28.9	2592.5±48.3

Cymodocea nodosa	Value			Trend	Test	P
Carbon (%)	23.78±6.89	31.89±4.08	38.98±3.58	increase	1	0.161
Nitrogen (%)	1.22±0.35	1.31±0.17	1.75±0.17	none	1	0.302
C:N ratio	19.02±0.69^a^	24.25±0.06^b^	22.25±0.20^ab^	intermediate	2	**<0.001**
δ^13^C	−11.42±0.03^a^	−11.68±0.05^ab^	−11.90±0.19^b^	decrease	2	**0.013**
δ^15^N	1.69±0.18^a^	0.13±0.04^b^	0.15±0.06^ab^	decrease	2	**0.013**
Lignin (%DM)^††^	3.84±0.06^a^	4.30±0.10^b^	5.70±0.16^c^	increase	1	**<0.001**

Average (±SE) temperature, salinity and pH were collected on different visits from Sept 2009 to May 2011 (n = 60). Total Alkalinity (TA) was calculated from water samples collected at each site on April and November 2010 (n = 4). Statistical analyses: 1, one-factor ANOVA with Holm-Sidak multiple comparisons; 2, Kruskal-Wallis One Way Analysis of Variance on Ranks with Tukey or Dunns multiple comparisons.^†^Carbonate chemistry previously published in Arnold et al 2012. ^††^Lignin analyses conducted by the Cumberland Valley Forage lab in Cumberland Co, Maryland using the methods of Goering and Van Soest (1970).

Values are means +/− SE.

**Table 3:** Composition of widgeon grass subjected to Free Ocean Carbon Enrichment within the St. Mary's River, Maryland (USA) in May-July 2010.

Conditions	Seawater carbonate chemistry^†^		
Distance from injector	500 cm	40 cm	5 cm
Temperature (C)	25.0	25.0	25.0
Salinity	17	17	17
pH	8.4	8.0	6.9
pCO_2_ (µtm)	157.8	469.3	6792.0
TA (µmol kg^−1^)	1467.0	1444.0	1455.0

Ruppia maritima	Value			Trend	Test	P
Carbon (%)	23.79±2.40	29.10±2.06	23.98±2.20	none	1	0.190
Nitrogen (%)	2.34±0.20	2.41±0.11	2.08±0.18	none	1	0.345
C:N ratio	10.24±0.93	12.21±1.16	11.57±0.77	none	1	0.406
δ^13^C	−13.20±0.26	−12.67±0.25	−12.82±0.20	none	1	0.296
δ^15^N	11.06±0.05	11.12±±0.08	10.93±0.06	none	1	0.129
Crude protein (%DM)	15.34±0.39	13.82±0.56	13.92±0.41	none	1	0.066
Adj. protein (%DM)	13.56±0.37	12.36±0.66	12.26±0.42	none	1	0.167
Starch (%DM)	3.08±0.77	4.00±0.82	3.76±0.70	none	1	0.684
Sugar (%DM)	9.14±2.12	10.40±0.90	8.70±1.62	none	1	0.750
Lignin (%DM)^††^	12.60±0.62^a^	15.67±0.57^b^	15.25±1.11^ab^	increase	1	**0.027**

Statistical analyses: 1, one-factor ANOVA with Holm-Sidak multiple comparisons. Letters indicate results of pairwise comparisons test *P*<0.05. ^†^Carbonate chemistry previously published in Arnold et al 2012. ^††^Lignin analyses conducted by the Cumberland Valley Forage lab in Cumberland Co, Maryland using the methods of Goering and Van Soest (1970).

Values are means +/− SE.

In contrast the secondary chemistry of *Z. muelleri* near Myora Springs was dramatically different (Fig. 3). Levels of Folin-reactive phenolics were reduced 87% in leaf tissues of these plants, compared to those located 30–50 m away. Condensed tannins, normally present at relatively high concentrations (15.5% of seagrass wet mass), were undetectable in leaf tissues collected near Myora Springs. Similarly, concentrations of phenolic acids decreased ≥93% with some compounds normally present in this species reduced to undetectable levels. In general, the phenolic metabolites of *Z. muelleri* responded to low pH conditions near Myora Springs in much the same way that other seagrass species respond to low pH and high CO_2_ conditions elsewhere. Previous studies revealed comparable losses of seagrass phenolics in *Cymodocea nodosa* and *Posidonia* sp. near high CO_2_ vents in the Mediterranean Sea and *Ruppia maritima* and *Potamogeton perfoliatus* exposed to free ocean carbon enrichment in the Chesapeake Bay (USA) [12], [13].

We quantified leaf lignin contents because these polyphenols are also products of the SA/PP pathway [57] and can influence herbivore feeding behaviors and digestion efficiencies [58]. We hypothesized that concentrations of lignin, like those of the other SA/PP phenolics, would be reduced; however, surprisingly, we found that lignin concentrations of *Z. muelleri* were not affected by proximity to the spring (Fig. 3). To determine if this was a common occurrence we again analyzed stored tissues of *Cymodocea nodosa* and *Ruppia maritima* from our previous studies [12]. In these cases we observed significant *increases* in lignin in seagrasses exposed to low pH / high CO_2_ waters (Tables 2, 3). The lignin contents of seagrasses collected near a natural CO_2_ vent site and exposed to high CO_2_/low pH conditions in FOCE experiments in the Chesapeake Bay were 150% and 124% higher, respectively, than lignin contents of nearby seagrasses. The results of all three studies indicate that while levels of soluble phenolics were consistently reduced at the various low pH / high CO_2_ sites, the concentrations of lignin did not decrease. These observations would be familiar to those studying the response of terrestrial plants to high CO_2_; for example, in land plants exposed to elevated atmospheric CO_2_ concentrations in free air carbon enrichment studies lignin levels are often increased or unaffected, but are rarely reduced (e.g., [59]–[62]). For studies of aquatic plants, such as seagrasses, we must also consider the potential impact of seawater pH, irrespective of elevated CO_2_ availability. Low pH can trigger ‘acid growth’ which softens plant cell walls by stimulating the activity of pH-sensitive expansin enzymes and the expression of related genes [63], [64]. Expanded cell wall structures are subsequently stabilized [64], in part by acid-induced lignification [65]. Instances of enhanced lignin production, where they occur [12], could help to explain the depletion of phenolic acids pools, as some of these compounds are required precursors in lignin biosynthesis. This suggests a growth vs. defense tradeoff that would be difficult to untangle, given that many of these SA/PP compounds have multiple roles in plants [66].

Many marine grazers, including fish, turtles and dugongs, tend to prefer species with lower levels of neutral digestible fiber (a combination of lignins and cellulosic substances) [67]–[70]. However, since we did not observe altered lignin levels in the leaves of *Z. muelleri* here this would not explain the feeding preferences exhibited by the rabbitfish in our feeding trials. Rather the “per bite” nutritional quality of *Z. muelleri*, and the feeding behavior of grazing fish, is most likely to have been determined but by soluble phenolics. These compounds are the only characteristics of the food items shown to have changed significantly in response to spring effluent. This may explain the near-instantaneous food choices of *Siganus fuscescens* during feeding trials. We observed that fish seemed to select preferred food items using either visual or olfactory cues, perceiving differences we could not. They generally did not browse or taste multiple food items during feeding trials. We hypothesize that the changing phenolic chemistry of *Z. muelleri* was dramatic enough to be readily sensed by juvenile rabbitfish. Many fish and sea turtles have UV sensitive vision capable of detecting wavelengths of light absorbed strongly by plant phenolics, at least when young [71]–[73]. As fish mature UV sensitive cones are often modified and detect only blue light [71]–[72]. Interestingly, this is when rabbittfish lose their proclivity for consuming seagrasses.

Overall, our observations demonstrate the groundwater discharge at Myora Springs alters the phenolic qualities of nearby seagrasses and the feeding behavior of certain herbivores. Similar results were observed in previous studies examining seagrasses exposed to high CO_2_ / low pH conditions near natural vent sites and generated by a series of simplified FOCE experiments [12]. Those studies sought to simulate, as closely as possible, future conditions of ocean acidification. In contrast, the situation at the Myora Springs site, where the exposure to low pH conditions is intermittent, is probably not an accurate simulation of anthropogenic ocean acidification. Nevertheless, these are naturally-occurring low pH conditions, a type of “coastal acidification”, which may have existed at Myora Springs for at least the last 105,000 years [10] and is common at other coastal groundwater discharge sites. Based on these findings we would predict that such sites would be popular feeding grounds for seagrass grazers seeking to reduce their exposure to soluble phenolics.

## References

[1] CuttrisAK, PrinceJB, CastleyJG (2013) Seagrass communities in southern Moreton Bay, Australia: coverage and fragmentations trends between 1987 and 2005. Aq Bot 108: 41–47.

[2] YoungPC, KirkmanH (1975) The seagrass communities of Moreton Bay, Queensland. Aq Bot 1: 191–202.

[3] HagiharaR, JonesRE, GrechA, LanyonJM, SheppardJK, MarshH (2013) Improving population estimates by quantifying diving and surfacing patterns: A dugong example. Mar Mamm Sci 30(1): 348–366.

[4] LimpusCJ, CouperPJ, ReadMA (1994) The green turtle, *Chelonia mydas*, in Queensland: Population structure in a warm temperate feeding area. Memoirs of the Queensland Museum (35)1: 139–154.

[5] Lanyon J, Limpus C, Marsh H (1989) Dugongs and turtles: grazers in the seagrass system. In: Larkum A, Mccomb A, Shepherd S (eds) Biology of Seagrasses. pp: 610–634

[6] WengHT (1990) Fish in shallow areas in Moreton Bay, Queensland and factors affecting their distribution. Est Coast Shelf Sci 30(6): 569–578.

[7] LeachLM (2011) Hydrology and physical setting of North Stradbroke Island. Proc Royal Soc Queensland 133–140.

[8] Natural Resources and Water (2006) Hydrology of North Stradbroke Island. Queensland Government www.nrw.qld.gov.au.

[9] LaylockJT (1975) North Stradbroke Island – Hydrogeological Report. Rep. No. 88 Geol. Surv.Qld

[10] MossP, PetherickL, NeilD (2011) Environmental change at Myora Springs, North Stradbroke Island over the last millennium. Proc Royal Soc Queensland Pg 133–140.

[11] MartinS, et al (2008) Effects of naturally acidified seawater on seagrass calcareous epibionts. Biol Letters 4: 689–692.10.1098/rsbl.2008.0412PMC261417118782731

[12] ArnoldT, MealeyC, LeaheyH, MillerAW, Hall-SpencerJM, et al (2012) Ocean Acidification and the Loss of Phenolic Substances in Marine Plants. PLoS ONE 7(4): e35107 doi:10.1371/journal.pone.0035107 2255812010.1371/journal.pone.0035107PMC3338829

[13] Migliore L, Piccenna A, Rotini A, Garrard S, Cristina Buia M (2012) Can ocean acidification affect chemical defenses in *Posidonia oceanica*? Mediterranean Seagrass Workshop 2012 program

[14] LindrothR (2010) Impacts of Elevated Atmospheric CO_2_ and O_3_ on Forests: Phytochemistry, Trophic Interactions, and Ecosystem Dynamics. J Chem Ecol 36: 2–21.2005461910.1007/s10886-009-9731-4

[15] Bidart-BouzatMG, Imeh-NathanieA (2008) Global change effects on plant chemical defenses against insect herbivores. J Integr Plant Biol 50: 1339–1354.1901712210.1111/j.1744-7909.2008.00751.x

[16] ValkamaE, KorchevaJ, OksanenE (2007) Effects of elevated O_3_, alone and in combination with elevated CO_2_, on tree leaf chemistry and insect herbivore performance: a meta-analysis. Glob Change Biol 13: 184–201.

[17] ColeyPD, MassaM, LovelockCE, WinterK (2002) Effects of elevated CO_2_ on foliar chemistry of saplings of nine species of tropical tree. Oecologia 133: 62–69.2459937010.1007/s00442-002-1005-6

[18] PeňuelasJ, EstiarteM (1998) Can elevated CO_2_ affect secondary metabolism and ecosystem function? Trends Ecol Evol 13: 20–24.2123818010.1016/s0169-5347(97)01235-4

[19] PeňuelasJ, EstiarteM, LlusiaJ (1997) Carbon-based secondary compounds at elevated CO_2_ . Photosynthetica 33: 313–316.

[20] StilingP, CornelissenT (2007) How does elevated carbon dioxide (CO_2_) affect plant–herbivore interactions? A field experiment and meta-analysis of CO_2_-mediated changes on plant chemistry and herbivore performance. Glob Change Biol 13: 1823–1842.

[21] MeehamTD, CrossleyMS, LindrothRL (2010) Impacts of elevated CO_2_ and O_3_ on aspen leaf litter chemistry and earthworm and springtail productivity. Soil Biol Biochem 42 (7): 1132–113.

[22] BryantJP, ChapinFSIII, KleinDR (1983) Carbon/nutrient balance of boreal plants in relation to vertebrate herbivory. Oikos 40: 357–368.

[23] MattsonWJ, Julkunen-TiittoR, HermsDA (2005) CO_2_ enrichment and carbon partitioning to phenolics: do plant responses accord better with the protein competition or the growth-differentiation balance models? Oikos 111: 337–347.

[24] VogtT (2010) Phenylpropenoid biosynthesis. Mol Plant 3(1): 2–20.2003503710.1093/mp/ssp106

[25] ValielaI, KoumjianL, SwainT, TealJM, HobbieJE (1979) Cinnamic acid inhibition of detritus feeding. Nature 280: 55–57.

[26] HarrisonPG (1982) Control of microbial growth and of amphipod grazing by water-soluble com- pounds from the leaves of *Zostera marina* . Mar Biol 67: 225–230.

[27] ArnoldT, TargettN (2002) Marine tannins: the importance of a mechanistic framework for predicting ecological roles. J Chem Ecol 28: 1919–1934.1247489110.1023/a:1020737609151

[28] HarrisonPG, ChanAT (1980) Inhibition of the growth of micro-algae and bacteria by extracts of eelgrass (*Zostera marina*) leaves. Mar Biol 61: 21–26.

[29] HarrisonPG, DuranceC (1989) Reductions in photosynthetic carbon uptake in epiphytic diatoms by water-soluble extracts of leaves of *Zostera marina.* . Mar Biol 90: 117–119.

[30] RavnH, AndaryC, KovacsG, MolgaardP (1989) Caffeic acid esters as *in vivo* inhibitors of plant pathogenic bacteria and fungi. Biochem Syst Ecol 17: 175–184.

[31] VergeerLHT, AartsTL, De GrootJD (1995) The ‘wasting disease’ and the effect of abiotic factors (light intensity, temperature, salinity) and infection with *Labyrinthula zosterae* on the phenolic content of *Zostera marina* shoots. Aq Bot 52: 35–44.

[32] McMillanC (1984) The condensed tannins (proanthocyanidins) in seagrasses. Aq Bot 20: 351–357.

[33] QuackenbushRC, BunnD, LingrenW (1996) HPLC determination of phenolic acids in the water-soluble extract of *Zostera marina* L. (eelgrass) Aq Bot 24(1): 83–89.

[34] RavnH, PedersenMF, BorumJ, AndaryC, AnthoniU, ChristophersonC, NielsonPH (1994) Seasonal variation and distribution of two phenolic compounds, rosmarinic acid and caffeic acid, in leaves and roots-rhizomes of eelgrass (*Zostera marina* L. Ophelia 40: 51–61.

[35] MuehlsteinLK (1992) The host-pathogen interaction in the wasting disease of eelgrass, *Zostera marina.* . Can J Bot 70: 2081–2088.

[36] Den Hartog C (1996) Sudden declines of seagrass beds; “wasting disease” and other disasters in JKuo, R. CPhillips, K. IWalkers, and HKirkman (eds.). Seagrass Biology: Proceedings of an International Workshop, 25–29 January 1996, Rottnest Island, Western Austalia. pp. 307–315,

[37] VergeerLHT, DeveliA (1997) Phenolic acids in healthy and infected leaves of *Zostera marina* and their growth limiting properties towards *Labyrinthula zosterae.* . Aq Bot 58: 65–72.

[38] DicksonAG, Sabine CL &ChristianJR (2007) Guide to Best Practices for Ocean CO_2_ Measurements (PICES Special Publication 3, 2007); available at. http://cdiac.ornl.gov/oceans/Handbook_2007.html.

[39] PierrotDE, WallaceDW (2006) MS Excel Program Developed for CO_2_ System. Calculation ORNL/CDIAC-105a (Carbon Dioxide Information Analysis Center, 2006).

[40] CaiWJ, WangY (1998) The chemistry, fluxes, and sources of carbon dioxide in the estuarine waters of the Satilla and Althamaha Rivers, Georgia. Limnol Oceanogr 43: 657–668.

[41] PetersonCH, RenaudPE (1989) Analysis of feeding preference experiments. Oecologia 80: 82–86.2349434910.1007/BF00789935

[42] ZapataO, McMillianC (1979) Phenolic acids in seagrasses. Aq Bot 7: 307–317.

[43] SteeleL, CaldwellM, BoettcherA, ArnoldT (2005) Seagrass-pathogen interactions: ‘pseudo-induction’ of turtlegrass phenolics near wasting disease lesions. Mar Ecol Prog Ser 303: 123–131.

[44] Hagerman AE, Klucher KM (1986) Tannins-protein interactions. In: Plant Flavanoids in Biology and Medicine: Biochemical, Pharmacological and Structure-Activity Relationships, 1986, eds Cody V, Middleton E & Harborne J. Alan R Liss, New York, pp 67–76.

[45] ArnoldTM, AppelH, PatelV, StocumE, KavalierA, SchultzJC (2004) Carbohydrate translocation determines the phenolic content of *Populus* foliage: a test of the sink-source model of plant defense. New Phytol 164(1): 157–164.10.1111/j.1469-8137.2004.01157.x33873480

[46] ArnoldTM, TannerCE, HatchWI (1995) Polyphenolic concentration of *Lobophora variegata* as a function of nitrogen availability. Mar Ecol Progr Ser 123: 177–183.

[47] FosterCE, MartinTM, PaulyM (2010) Comprehensive Compositional Analysis of Plant Cell Walls (Lignocellulosic biomass) Part I: Lignin. Vis Exp 37, e1745, doi:10.3791/1745 10.3791/1745PMC314457620224547

[48] UdyJW, DennisonWC (1997) Physiological responses of seagrass used to identify anthropogenic nutrient inputs. Mar Freshwater Res 48: 605–614.

[49] PradoP, HeckK (2011) Seagrass selection by omnivorous and herbivorous consumers: determining factors. Mar Ecol Progr Ser 429: 45–55.

[50] GoeckerME, HeckKL, ValentineJF (2005) Effects of nitrogen concentrations in turtlegrass *Thalassia testudinum* on consumption by the bucktooth parrotfish *Sparisoma radians.* . Mar Ecol Progr Ser 286: 239–248.

[51] de los SantosCB, BrunFG, NonodaY, CambridgeML, BoumaTJ, VergaraJJ, Pérez-LlorénsJL (2012) Leaf-fracture properties correlated with nutritional traits in nine Australian seagrass species: implications for susceptibility to herbivory. Mar Ecol Prog Ser 458: 89–102.

[52] TomasF, AbbottJM, SteinbergC, BalkM, WilliamsSL, StachowiczJJ (2011) Plant genotype and nitrogen loading influence seagrass productivity, biochemistry, and plant–herbivore interactions. Ecology 92(9): 1807–1817.2193907710.1890/10-2095.1

[53] GriceAM, LoneraganNR, DennisonWC (1996) Light intensity and the interactions between physiology, morphology, and stable isotope ratios in five species of seagrass. J Exp Mar Biol Ecol 195: 91–110.

[54] BeerS, RehnbergJ (1997) The acquisition of inorganic carbon by the seagrass *Zostera marina* . Aq Bot 56: 277–283.

[55] BeerS, KochE (1996) Photosynthesis of marine macroalgae and seagrasses in globally changing CO_2_ environments. Mar Ecol Progr Ser 141 (1–3): 199–204.

[56] VizziniS, et al (2010) Effect of explosive shallow hydrothermal vents on δ^13^C and growth performance in the seagrass *Posidonia oceanica* . J Ecol 98: 1284–1291.

[57] DixonRA, et al (2002) The phenylpropanoid pathway and plant defence—a genomics perspective. Mol Plant Path 3(5): 371–390.2056934410.1046/j.1364-3703.2002.00131.x

[58] VergesA, BecerroMA, AlcoverroT, RomeroJ (2007) Experimental evidence of chemical deterrence against multiple herbivores in the seagrass *Posidonia oceanica.* . Mar Ecol Progr Ser 343: 107–114.

[59] LuoZ-B, PolleA (2009) Wood composition and energy content in a poplar short rotation plantation on fertilized agricultural land in a future CO_2_ atmosphere. Glob Change Biol 15(1): 38–47.

[60] CsekeLJ, TsaiC-J, RogersA, et al (2009) Transcriptomic comparison in the leaves of two aspen genotypes having similar carbon assimilation rates but different partitioning patterns under elevated CO_2_ . New Phytol 182(4): 891–911.1938309810.1111/j.1469-8137.2009.02812.x

[61] LuoZ-B, CalfapietraC, Scarascia-MugnozzaG (2008) Carbon-based secondary metabolites and internal nitrogen pools in *Populus nigra* under Free Air CO_2_ Enrichment (FACE) and nitrogen fertilization. Plant Soil 304(1–2): 45–57.

[62] AkinDE, KimballBA, WindhamWR, et al (1995) Effect of free-air CO_2_ enrichment (FACE) on forage quality of wheat. Anim Feed Sci Tech 53(1): 29–43.

[63] CosgroveDJ (1999) Enzymes and other agents that enhance cell wall extensibility. Annu. Rev. Plant Physiol. Plant Mol Biol 50: 391–417.10.1146/annurev.arplant.50.1.39111541953

[64] LagerI, AndreassonO, DunbarTL, et al (2010) Changes in external pH rapidly alter plant gene expression and modulate auxin and elicitor responses. Plant Cell Env 33(9): 1513–1528.2044421610.1111/j.1365-3040.2010.02161.xPMC2920358

[65] GrabberJH, HatfieldRD, RalphJ (2003) Apoplastic pH and monolignol addition rate effects on lignin formation and cell wall degradability in maize. J Agric Food Chem 51: 4984–4989.1290395710.1021/jf030027c

[66] HermsDA, MattsonWJ (1992) The dilemma of plants – to grow or defend. Q Rev Biol 67: 283–335.

[67] MarianiS, AlcoverroT (1999) A multiple-choice feeding-preference experiments utilizing seagrasses with a natural population of herbivorous fishes. Mar Ecol Progr Ser 189: 295–299.

[68] PreenA (1995) Impacts of dugong foraging on seagrass habitats: observational and experimental evidence for cultivation grazing. Mar Ecol Prog Ser 124: 201–213.

[69] Lanyon JM, Limpus CJ, Marsh H (1989) Dugongs and turtles: grazers in the seagrass system. In: Larkum AWD, McComb AJ, Shepherd SA (eds) Biology of seagrasses. A treatise on the biology of seagrasses with special reference to the Australian Region. Aquatic plant studies 2. Elsevier, Amsterdam, p 610–634

[70] Brand-GardnerSJ, LanyonJM, LimpusCJ (1999) Diet selection by immature green turtles, *Chelonia mydas*, in subtropical, Moreton Bay, south-east Queensland. Aus J Zool 47: 181–191.

[71] LoseyGS, CroninTW, GoldsmithTH, HydesD, MarshallNJ, McFarlandWN (1998) The UV visual world of fishes: a review. J Fish Biol 54: 921–943.

[72] FlamariqueIN (2012) Opsin switch reveals function of the ultraviolet cone in fish foraging. Proc Royal Soc 280: 20122490.10.1098/rspb.2012.2490PMC357430923222448

[73] MähergerLM, LitherlandL, FritchesKA (2007) An anatomical study of the visual capabilities of the green turtle, *Chelonia mydas* . Copea 1: 169–179.

